The article "Tranexamic Acid in Pregnant Women With Placenta Previa: A Double-Blind, Multicenter Randomized Clinical Trial" was retracted in 2025. Reasons: original data or images not available; unreliable results or conclusions; concerns about the article.

# Tranexamic Acid in Pregnant Women With Placenta Previa: A Double-Blind, Multicenter Randomized Clinical Trial

**DOI:** 10.7759/cureus.75297

**Published:** 2024-12-07

**Authors:** Shahla Alalaf, Ariana K Jawad, Namir G Al-Tawil, Kawa F Dizaye, Sileem A Sileem, Noor Elebiary, Zanwer S Mahmood, Rozhan Y Khalil, Khalida M Amin, Nazdaar R Ali

**Affiliations:** 1 Obstetrics and Gynecology, Hawler Medical University, College of Medicine, Erbil, IRQ; 2 Obstetrics and Gynecology, Kurdistan Higher Council of Medical Specialties, Erbil, IRQ; 3 Community Medicine, Hawler Medical University, Erbil, IRQ; 4 Pharmacology, Hawler Medical University, College of Medicine, Erbil, IRQ; 5 Obstetrics and Gynecology, Al-Azhar University, Faculty of Medicine, Assuit, EGY; 6 Obstetrics and Gynecology, Ninewells Hospital, Dundee, GBR; 7 Obstetrics and Gynecology, Ministry of Health, Maternity Teaching Hospital, Erbil, IRQ; 8 Obstetrics and Gynecology, College of Medicine, University of Sulaimani, Sulaimaniyah, IRQ; 9 Obstetrics and Gynecology, University of Kirkuk, Kirkuk Medical College, Kirkuk, IRQ; 10 Obstetrics and Gynecology, Duhok Obstetrics and Gynecology Teaching Hospital, Duhok, IRQ

**Keywords:** intravenous tranexamic acid, perinatal mortality, placenta previa, preterm labour, stillbirth

## Abstract

Aims: To determine the effectiveness of tranexamic acid (TXA) in reducing vaginal bleeding, extending pregnancy duration, and enhancing perinatal outcomes in pregnant women with placenta previa.

Methods: A multicenter, randomized, double-blind clinical trial was conducted at three maternity teaching hospitals in Iraq's Kurdistan region, Azadi Hospital in the north of Iraq, and Al-Azhar University Hospital in Egypt on 146 women with placenta previa. Participants were randomly assigned to two interventional groups in a 1:1 ratio to receive either TXA or Dextrose 5% water (D5W). The two groups were compared in terms of the cessation of vaginal bleeding, continuation of pregnancy to term, and the perinatal outcome after repeated use of either method of treatment.

Results: Bleeding stopped in 91.8% of the TXA group; however, the placebo group had more admissions for blood transfusion, received more units of packed red blood cells, and almost all their deliveries were preterm compared with the TXA group. Factors significantly associated with ‘stopped bleeding’ were TXA (OR = 5.2; 95% CI = 1.7-15.5), BMI of < 25 kg/m^2^ (OR = 6.3; 95% CI = 1.2-35.5), and BMI of 25-29 kg/m^2^, late preterm delivery (32-36+6 weeks) [OR = 20.6; 95% CI = 4.6-90.2], and term delivery (39-40+6 weeks) [OR = 4.5; 95% CI = 4.5-776.2] compared with very preterm deliveries (28-32+6 weeks).

Conclusions: Treatment with TXA during pregnancy in women with placenta previa significantly outperforms in managing vaginal bleeding, prolonging pregnancy to a favorable gestational age and perinatal outcome. Larger studies are needed to confirm its benefits and guide clinical practice.

The article "Tranexamic Acid in Pregnant Women With Placenta Previa: A Double-Blind, Multicenter Randomized Clinical Trial" was retracted in 2025. Reasons: original data or images not available; unreliable results or conclusions; concerns about the article.

## Introduction

Placenta previa is a serious obstetric complication, occurring in approximately 0.5% of pregnancies [1]. It is associated with significant maternal and perinatal morbidity and mortality [2], and its management remains challenging [3].

Significant vaginal hemorrhage, regardless of the cause, necessitates an urgent assessment of maternal and fetal status, fluid resuscitation, blood product transfusion as indicated, and timely delivery if the bleeding does not subside, irrespective of gestational age, even if the gestation is preterm [4]. Preterm delivery due to excessive vaginal bleeding increases the risk of perinatal mortality, lower birth weight, lower Appearance, Pulse, Grimace, Activity, and Respiration (APGAR) scores, and respiratory distress syndrome [5].

Furthermore, vaginal bleeding due to placenta previa is associated with increased maternal morbidity. This condition can result in significant blood loss, necessitating blood transfusion, and potentially leading to postpartum hemorrhage (PPH), anemia, and cesarean hysterectomy, depending on the severity and location of the placenta [6]. Although various management strategies are available depending on the severity of the presentation, definitive treatment for placenta previa remains unavailable [7]. Currently, expectant management is employed for placenta previa, and the guidelines primarily focus on the mode and timing of delivery and supportive maternal and fetal well-being during hospital admission and monitoring [8]. Data on the use of interventional medications for placenta previa are limited and mostly inconsistent, rendering their overall effectiveness inconclusive [9].

Tranexamic acid (TXA) is an antifibrinolytic agent that reduces blood loss and transfusion requirements under various medical, surgical, and gynecological conditions [10].

A meta-analysis of 18 randomized controlled trials reported beneficial effects of TXA in reducing blood loss and blood transfusion requirements in pregnant women undergoing CS, demonstrating its effectiveness in successfully reducing blood loss during these procedures [11].

Human trials of TXA use in pregnancies complicated by placenta previa remain lacking. Furthermore, although TXA has been recognized as a category B drug during pregnancy [12], its safety and effectiveness in managing women with placenta previa have not been well studied.

We hypothesized that TXA would be safe during pregnancy and decrease the recurrence of vaginal bleeding in women with placenta previa. Accordingly, this study aimed to determine the effectiveness of TXA as an interventional drug for decreasing vaginal blood loss and prolonging pregnancy in women with placenta previa, thereby improving perinatal outcomes.

The article "Tranexamic Acid in Pregnant Women With Placenta Previa: A Double-Blind, Multicenter Randomized Clinical Trial" was retracted in 2025. Reasons: original data or images not available; unreliable results or conclusions; concerns about the article.

## Materials and methods

Study design and setting

This multicenter, randomized, double-blind clinical trial was conducted at the Maternity Teaching Hospital in Erbil City, Sulaimani Maternity Teaching Hospital, and Duhok Obstetrics and Gynecology Teaching Hospital, all located in the Kurdistan region of Iraq; Azadi Teaching Hospital in Kirkuk City, north Iraq; and Al-Azhar University Hospital in Assuit City, Egypt. These public hospitals are recognized for their high annual delivery rates and provide 24-hour services to a diverse population of pregnant women, including those with high-risk pregnancies. The participant recruitment and follow-up in this study were conducted from December 10, 2022, to December 3, 2023.

Eligibility criteria

Ethical clearance was obtained from the research ethics committees, and 146 pregnant women of all parties with placenta previa were included in the trial based on the following inclusion criteria: gestation age of ≥28 weeks, recurrent episodes of painless vaginal bleeding that either flooded underwear or required the use of a pad, bleeding due to placenta previa, hemodynamically stable, and willingness to participate in the trial. Women with placenta previa and accreta, those who presented with severe vaginal bleeding and abdominal pain, those who were hemodynamically unstable, those with fetal distress that required immediate intervention, those with contraindications to the use of TXA (hypersensitivity, acquired defective color vision, history of venous thromboembolism), those with preexisting medical conditions that could potentially affect the outcome of the pregnancy (e.g., diabetes mellitus, preeclampsia, heart disease, renal illness), smokers, and those who declined to participate in the trial were excluded from the study.

Definition, diagnostic criteria, and grading classifications of placenta previa

Placenta previa was defined as the presence of a lowly positioned placenta in the lower uterine segment. It was diagnosed using ultrasonography (US) performed by experienced sonographers at each hospital. The transabdominal US, followed by transvaginal US assessment, was used to determine the placental location. Based on the distance of the placental edge from the internal cervical os, placenta previa was categorized into the following three groups:

Marginal placenta previa: the distance between the placental edge and the internal cervical os is <2 cm. Partial placenta previa: the lower edge of the placenta partially overlaps with the internal cervical os. Complete placenta previa: the placenta completely overlaps the internal cervical os [13].

The article "Tranexamic Acid in Pregnant Women With Placenta Previa: A Double-Blind, Multicenter Randomized Clinical Trial" was retracted in 2025. Reasons: original data or images not available; unreliable results or conclusions; concerns about the article.

Furthermore, US was used to determine the placental edge (including the thickness and presence of a marginal sinus) and associated findings that may reveal placenta accrete.

Randomization and blinding

A total of 149 participants were randomly assigned to two groups in a 1:1 ratio by a statistician at the College of Medicine, who was blinded to the research purposes, using a random allocation software program (version 2.0) [14]. The participants receive either TXA or Dextrose 5% in water (D5W). Notably, participants were divided into two groups using block randomization, with 75 participants in one group and 74 in the other.

After preparing a random sequence, women were allocated to two trial groups using numbered containers with the same sequences applied in the randomization process. These numbers were allocated to the containers by an individual blinded to the research protocol (the encoder). Each participant was assigned a unique identification (UI) code during allocation. The same code was used for repeated hospital admissions, ensuring that the patients received the same intervention each time. Identical 30-mL disposable syringes were used in both groups, which were visually indistinguishable (same color, shape, and size), except for unique UI labels that concealed the patient group from the primary researchers. After completion of the trial, the UIs were decoded to determine the participant group. The primary researchers who conducted the interventions in each of the five hospitals were provided with UI containers daily throughout the study period.

Individual participant data from this trial were added to the clinical electronic notes. All participating centers approved the study protocol. Any queries and progress regarding individual cases were discussed between the study leads in each of the abovementioned centers.

Sample size estimation

The sample size was estimated using Power and Sample Size Calculation software (version 3.0.43). First, we conducted a pilot study with two groups of 10 women, each involving the same study design and follow-up as in the present study, owing to the lack of published studies on the efficacy of TXA in reducing vaginal blood loss in women with placenta previa. Statistical power analysis was performed using two different success rates: 90% for the TXA group and 70% for the control group. Finally, a total sample size of 140 women (70 per group) was estimated with a significance level of 0.05 and a power of 85%.

The article "Tranexamic Acid in Pregnant Women With Placenta Previa: A Double-Blind, Multicenter Randomized Clinical Trial" was retracted in 2025. Reasons: original data or images not available; unreliable results or conclusions; concerns about the article.

Participant grouping

A total of 188 pregnant women with placenta previa were assessed for eligibility in five hospital settings during the study period. Notably, 39 women were excluded because they either did not meet the recruitment criteria or refused to participate. Randomization of the two arms included 149 women, with 75 women in the TXA group and 74 in the placebo group. In the TXA group, two participants were lost to follow-up and were excluded from the analysis. In the placebo group, one woman was lost to follow-up. Finally, 73 women were included in each group. Figure 1 presents a flowchart outlining the participant recruitment process, trial design, and procedures following the CONSORT recommendations [15].

**Figure 1:** CONSORT Flowchart illustrating participant enrollment, allocation, follow-up, and analysis in the clinical trial

Interventions

Tranexamic Acid

The intervention group received 1 g TXA (2 ampules each of 500 mg/5 mL solution; Trenaxa; Macleods Pharmaceuticals Pvt. Ltd., Mumbai, India) diluted in 20 mL glucose water administered intravenously slowly twice daily for 48 h during each vaginal bleeding episode, along with standard expectant management. Each hospital admission was assigned a unique IU code.

*Dextrose 5% Water* 

The placebo group received 30 mL of Dextrose 5% water intravenously twice daily for 48 hours during each bleeding episode, along with standard expectant management. Each hospital admission was assigned a unique IU code.

Clinical Trial Outcome

The primary outcomes were as follows: (1) Hemostasis: Complete or gradual cessation of vaginal bleeding with repeated administration of both interventions. (2) Pregnancy reaching term: gestation of ≥37 weeks following TXA or placebo intervention. (3) Favorable perinatal outcomes: a viable newborn with a birth weight ≥2500 g, an APGAR score of ≥7, and no hospitalization to the neonatal intensive care unit (NICU).

The secondary outcomes were the frequency of hospital admissions and the need for blood transfusions.

Hospital Monitoring Strategies

Following each episode of vaginal bleeding, women were admitted to the hospital, and a comprehensive monitoring protocol was implemented to ensure the safety and efficacy of the TXA intervention. The monitoring strategies were the same in all trial centers, including monitoring of vital signs, assessment of vaginal bleeding (severity and amount of vaginal bleeding, with documentation of any changes), and regular monitoring of fetal well-being. Urine output was assessed to monitor renal function. Additionally, consultations with other specialists (e.g., hematologists and perinatologists) were offered according to specific care requirements. Follow-up visits were scheduled biweekly, with more frequent appointments as needed, to monitor maternal and fetal health.

The article "Tranexamic Acid in Pregnant Women With Placenta Previa: A Double-Blind, Multicenter Randomized Clinical Trial" was retracted in 2025. Reasons: original data or images not available; unreliable results or conclusions; concerns about the article.

Laboratory tests, including regular hemoglobin and hematocrit measurements, were performed during each hospital admission to monitor anemia. In addition, other relevant tests, such as coagulation profile, were conducted to evaluate blood loss and clotting status, as indicated, and blood-product transfusions were performed to manage acute blood loss. Corticosteroids were administered when preterm delivery was planned because of maternal or fetal reasons.

Scheduled Delivery

The timing of cesarean section (CS) was determined based on gestational age, fetal well-being, and severity of maternal bleeding, with the aim of achieving delivery at approximately 38-39 weeks. However, emergency CSs were performed in cases of life-threatening maternal hemorrhage or non-reassuring fetal status. Newborns received comprehensive pediatric monitoring from birth to discharge to ensure their well-being prior to leaving the hospital.

Data Collection

Demographic data, including participants' age, parity, and gestational age at the time of admission, confirmed using a first-trimester ultrasound at 11-14 weeks of gestation, were collected [16]. Body mass index (BMI) was calculated using a woman's pre-pregnancy or early first-trimester weight and was categorized as normal (BMI ≥18.5-24.9 kg/m^2^), overweight (BMI ≥25-29.9 kg/m^2^), and obese (BMI ≥30 kg/m^2^) [17].

The frequency of hospital admissions was documented, and vaginal bleeding was assessed as either having not stopped or gradually subsided with repeated interventions. The need for blood transfusion was also monitored based on the degree of vaginal bleeding, clinical evaluation of the mother's condition, and hemoglobin and hematocrit levels, and the total number of packed red blood cells (PRBCs) was recorded. Furthermore, the mode of delivery, elective CS, emergency CS, or vaginal, was recorded. Notably, vaginal delivery was the predominant mode of delivery in macerated stillbirths, contingent upon placental assessment.

Neonatal data, including fetal viability, admission to the NICU, and APGAR scores at 1 and 5 min (categorized as low [score ≤3], moderate [score 4-6], or reassuring [score ≥7], were collected [18]. Gestational age was categorized into five groups: very preterm (28-31 + 6 weeks), moderate to late preterm (32-36 + 6 weeks), early term (37-38 + 6 weeks), and full-term (39-40 + 6 weeks) [19,20]. Notably, a discrepancy between the gestational age at delivery and that at the time of initial admission was reported. Birth weight was classified into four groups: extremely low (<1000 g), very low (1000-1499 g), low (1500-2499 g), and normal (2500-3999 g) [21,22].

The article "Tranexamic Acid in Pregnant Women With Placenta Previa: A Double-Blind, Multicenter Randomized Clinical Trial" was retracted in 2025. Reasons: original data or images not available; unreliable results or conclusions; concerns about the article.

Data Collection Methods

Data collection commenced with paper-based forms coded with IU by research staff trained in data collection procedures during the first interview with the patients. Subsequently, data were extracted from electronic health records. The individual responsible for data collection was blinded to the research purpose and the UI codes.

*Data and Safety Monitoring* 

An independent statistician with expertise in statistics, safety monitoring, and clinical trial requirements performed data entry. The data were evaluated regularly to monitor participant outcomes, safety, and the impact of interventions, as well as to evaluate the performance in achieving the study objectives.

An independent adjudication committee was formed to standardize the assessment of the primary and secondary outcomes. The committee consisted of two blinded specialists in obstetrics and gynecology with experience in clinical trials. They reviewed the data of the individual participants and applied predefined criteria to adjudicate the outcomes. Furthermore, a separate adjudication committee involving two hospital-affiliated, blinded obstetricians with experience in clinical trials was established to standardize the evaluation of the primary and secondary outcomes. They evaluated data from each participant and determined the results using predetermined standards.

Ethical Approval

This research was approved by the Research Ethics Committee/College of Medicine/Hawler Medical University (Nb.9/10 on September 11, 2022), which covered the four research settings in Iraq, and the Institutional Review Board/Al-Azhar-Assiut-Faculty of Medicine (AZAST/RESEARCH/52/7-SEP-2022) approved one research setting in Egypt. In addition, the institutional review board of each participating hospital approved the proposal before recruiting participants. This study was conducted in accordance with the ethical standards outlined in the Declaration of Helsinki. Participants provided written informed consent after receiving comprehensive information about the study, including their right to withdraw from the study at any time without any consequences. This study was prospectively registered on Clinical Trials (NCT05688111) on January 18, 2023, prior to conducting the research [31].

Statistical Analysis

Data were analyzed using IBM Corp. Released 2019. IBM SPSS Statistics for Windows, Version 26.0. Armonk, NY: IBM Corp. The student’s t-test (unpaired t-test) was used to compare the means of the two study groups. The Chi-square test of association was used to compare proportions. However, Fisher’s exact test was used instead of the chi-square test when the expected count (frequency) of >20% of the cells in the table was <5. Logistic regression analysis was used when the dependent variable was a binary categorical variable (such as bleeding stopped). Variables that showed significant associations with the dependent variables in univariate analysis were included in the regression model as independent variables. Statistical significance was set at p < 0.05.

The article "Tranexamic Acid in Pregnant Women With Placenta Previa: A Double-Blind, Multicenter Randomized Clinical Trial" was retracted in 2025. Reasons: original data or images not available; unreliable results or conclusions; concerns about the article.

## Results

In total, 146 women participated in this study, of which 73 received TXA and 73 received D5W. No significant differences were observed in age distribution, gestational age at first admission to the hospital, hospital admission, or BMI between the groups. However, a greater number of hospital admissions for blood transfusions and PRBC units were reported in the placebo group than in the TXA group (Table 1).

**Table 1:** Hospital admissions for both study populations *Calculated by Fisher’s exact test. A p-value of < 0.05 is considered significant

	Tranexamic acid	Glucose water	Total	Test statistics	p-value*
	No. (%)	No. (%)	No. (%)		
Admissions to the hospital till delivery					
1	46 (63.0)	35 (47.9)	81 (55.5)		
2	16 (21.9)	26 (35.6)	42 (28.8)		
3	9 (12.3)	10 (13.7)	19 (13.0)		
4	2 (2.7)	1 (1.4)	3 (2.1)		
5	0 (0.0)	1 (1.4)	1 (0.7)	5.264	0.216
No. of admissions for blood transfusion					
0	43 (58.9)	8 (11.0)	51 (34.9)		
1	17 (23.3)	38 (52.1)	55 (37.7)		
2	13 (17.8)	19 (26.0)	32 (21.9)		
3	0 (0.0)	6 (8.2)	6 (4.1)		
5	0 (0.0)	1 (1.4)	1 (0.7)		
6	0 (0.0)	1 (1.4)	1 (0.7)	42.905	<0.001
Pints of blood received					
0	43 (58.9)	8 (11.0)	51 (34.9)		
1	16 (21.9)	21 (28.8)	37 (25.3)		
2	8 (11.0)	26 (35.6)	34 (23.3)		
3	6 (8.2)	15 (20.5)	21 (14.3)		
4	0 (0.0)	1 (1.4)	1 (0.7)		
5	0 (0.0)	1 (1.4)	1 (0.7)		
6	0 (0.0)	1 (1.4)	1 (0.7)	42.788	<0.001
Total	73 (100.0)	73 (100.0)	146 (100.0)		

TXA was significantly more effective than glucose water in stopping vaginal bleeding. CSs constituted the majority of deliveries in both groups. Women in the TXA group were more likely to have live, normal-weight newborns with normal APGAR scores. Almost all (97.3%) deliveries in the placebo group were preterm compared with 75.3% in the TA (Table 2).

**Table 2:** Treatment outcomes in both study populations. *Calculated by Chi-square test. **Calculated by Fisher’s exact test. A p-value of < 0.05 is considered significant. CS: Cesarean section. NICU: Neonatal intensive care unit

	Tranexamic acid	Glucose water	Total	Test statistics	p-value
	No. (%)	No. (%)	No. (%)		
Response to treatment outcome					
Bleeding didn't stop	6 (8.2)	34 (46.6)	40 (27.4)		
Bleeding stopped	67 (91.8)	39 (53.4)	106 (72.6)	26.996	<0.001*
Mode of delivery					
Spontaneous vaginal delivery	4 (5.5)	3 (4.1)	7 (4.8)		
Elective C/S	45 (61.6)	38 (52.1)	83 (56.8)		
Emergency C/S	24 (32.9)	32 (43.8)	56 (38.4)	1.918	0.402**
Fetal outcome					
Fresh stillbirth	0 (0.0)	4 (5.5)	4 (2.7)		
Macerated stillbirth	0 (0.0)	1 (1.4)	1 (0.7)		
Alive with a normal APGAR score	67 (91.8)	31 (42.5)	98 (67.1)		
Low APGAR score with admission to NICU	3 (4.1)	31 (42.5)	34 (23.3)		
Early neonatal death	3 (4.1)	6 (8.2)	9 (6.2)	44.768	<0.001**
APGAR 1^st^ minute					
Low	3 (4.1)	13 (17.8)	16 (11.0)		
Moderately abnormal	12 (16.4)	38 (52.1)	50 (34.2)		
Reassuring	58 (79.5)	22 (30.1)	80 (54.8)	35.970	<0.001*
APGAR 5^th^ minute					
Low	2 (2.7)	12 (16.4)	14 (9.6)		
Moderately abnormal	3 (4.1)	22 (30.1)	25 (17.1)		
Reassuring	68 (93.2)	39 (53.4)	107 (73.3)	29.443	<0.001*
Gestational age at delivery					
Very preterm	2 (2.7)	19 (26.0)	21 (14.4)		
Late preterm	53 (72.6)	52 (71.2)	105 (71.9)		
Term	18 (24.7)	2 (2.7)	20 (13.7)	26.571	<0.001*
Low birth weight (LBW)					
Very LBW	2 (2.7)	8 (11.0)	10 (6.8)		
LBW	6 (8.2)	29 (39.7)	35 (24.0)		
Normal birth weight	65 (89.0)	36 (49.3)	101 (69.2)	27.041	<0.001*
Total	73 (100.0)	73 (100.0)	146 (100.0)		

The mean difference between gestational age at delivery and gestational age at first hospital admission was 5.6 and 1.7 weeks in the TXA and placebo groups, respectively (Figure 2).

The article "Tranexamic Acid in Pregnant Women With Placenta Previa: A Double-Blind, Multicenter Randomized Clinical Trial" was retracted in 2025. Reasons: original data or images not available; unreliable results or conclusions; concerns about the article.

**Figure 2:** Mean of difference between gestational age at delivery and at first visit among women of the two study groups. *Calculated by subtracting the gestational age at first visit from the gestational age at delivery. A p-value of < 0.05 is considered significant.

The factors associated with cessation of bleeding in both groups were the use of TXA, BMI, and term pregnancies (Table 3). 

**Table 3:** Predicting bleeding control in study population. *Calculated by Chi-square test. A p-value of < 0.05 is considered significant. BMI: Body mass index

	Bleeding stopped	Bleeding didn't stop	Total	Test statistics	p-value*
	No. (%)	No. (%)	No. (%)		
Intervention					
Tranexamic acid	67 (91.8)	6 (8.2)	73 (100.0)		
Glucose water	39 (53.4)	34 (46.6)	73 (100.0)	26.996	<0.001
Age (years)					
<20	5 (71.4)	2 (28.6)	7 (100.0)		
20-34	71 (76.3)	22 (23.7)	93 (100.0)		
≥ 35	30 (65.2)	16 (34.8)	46 (100.0)	1.921	0.383
BMI (Kg/m^2^)					
<25	18 (81.8)	4 (18.2)	22 (100.0)		
25-29	47 (83.9)	9 (16.1)	56 (100.0)		
≥ 30	40 (59.7)	27 (40.3)	67 (100.0)	10.111	0.006
Parity					
Primiparous	15 (83.3)	3 (16.7)	18 (100.0)		
Multiparous	53 (75.7)	17 (24.3)	70 (100.0)		
Grand Multiparous	38 (65.5)	20 (34.5)	58 (100.0)	2.847	0.241
Gestational age at delivery					
Very preterm	3 (14.3)	18 (85.7)	21 (100.0)		
Late preterm	84 (80.0)	21 (20.0)	105 (100.0)		
Term	19 (95.0)	1 (5.0)	20 (100.0)	43.837	<0.001
Total	106 (72.6)	40 (27.4)	146 (100.0)		

However, no significant association was observed between the degree of placenta previa and bleeding, preterm delivery, or fetal outcomes in women who received TXA. Similarly, these associations were not statistically significant in the placebo group (Table 4).

The article "Tranexamic Acid in Pregnant Women With Placenta Previa: A Double-Blind, Multicenter Randomized Clinical Trial" was retracted in 2025. Reasons: original data or images not available; unreliable results or conclusions; concerns about the article.

**Table 4:** Perinatal outcome by grades of placenta. *Calculated by Chi-square test. **Calculated by Fisher’s exact test. A p-value of < 0.05 is considered significant.  CS: Cesarean section. NICU: Neonatal intensive care unit

	Grades of placenta previa					
	Marginal	Partial	Complete	Total	Test statistics	p-value*
	No. (%)	No. (%)	No. (%)	No. (%)		
Tranexamic acid group						
Response to bleeding						
Bleeding stopped	44 (91.7)	19 (95.0)	4 (80.0)	67 (91.8)		
The bleeding didn't stop	4 (8.3)	1 (5.0)	1 (20.0)	6 (8.2)	1.645	0.466
GA at delivery						
Preterm	31 (64.6)	19 (95.0)	5 (100.0)	55 (75.3)		
Term	17 (35.4)	1 (5.0)	0 (0.0)	18 (24.7)	8.452	0.011
Fetal outcome						
Alive with a Normal APGAR Score	45 (93.8)	19 (95.0)	3 (60.0)	67 (91.8)		
Low APGAR score with Admission to NICU	2 (4.2)	0 (0.0)	1 (20.0)	3 (4.1)		
Early Neonatal Death	1 (2.1)	1 (5.0)	1 (20.0.)	3 (4.1)	7.416	0.092
Total	48 (100.0)	20 (100.0)	5 (100.0)	73 (100.0)		
Glucose water group						
Response to bleeding						
Bleeding stopped	27 (60.0)	11 (44.0)	1 (33.3)	39 (53.4)		
The bleeding didn't stop	18 (40.0)	14 (56.0)	2 (66.7)	34 (46.6)	2.226	0.376
GA at delivery						
Preterm	43 (95.6)	25 (100.0)	3 (100.0)	71 (97.3)		
Term	2 (4.4)	0 (0.0)	0 (0.0)	2 (2.7)	1.693	0.572
Fetal outcome						
FSB	2 (4.4)	2 (8.0)	0 (0.0)	4 (5.5)		
MSB	1 (2.2)	0 (0.0)	0 (0.0)	1 (1.4)		
Alive with a normal APGAR Score	23 (51.1)	8 (32.0)	0 (0.0)	31 (42.5)		
Low APGAR Score with admission to NICU	14 (31.1)	14 (56.0)	3 (100.0)	31 (42.5)		
Early Neonatal Death	5 (11.1)	1 (4.0)	0 (0.0)	6 (8.2)	10.709	0.202
Total	45 (100.0)	25 (100.0)	3 (100.0)	73 (100.0)		

The factors significantly associated with “stopped bleeding” were TXA (odds ratio [OR] = 5.2; 95% confidence interval [CI] = 1.7-15.5), BMI of <25 kg/m^2^ (OR = 6.3; 95% CI = 1.2-35.5), BMI of 25-29 kg/m^2^, late preterm delivery (OR = 20.6; 95% CI = 4.6-90.2), and term delivery (OR = 4.5; 95% CI = 4.5-776.2) (Table 5).

**Table 5:** SPSS output for binary logistic regression analysis where the dependent variable was stopped bleeding. ⁋B: regression coefficient. †Odds ratio. ††Confidence interval. A p-value of < 0.05 is considered significant. BMI: Body mass index

				95% CI of OR†	
	B^⁋^	p	OR^††^	Lower	Upper
Intervention					
Tranexamic acid	1.656	0.003	5.239	1.770	15.509
Glucose water (Reference)					
BMI (Kg/m^2^)		0.021			
< 25	1.856	0.034	6.398	1.152	35.549
25-29	1.228	0.025	3.416	1.168	9.985
≥ 30 (reference)					
Gestational age at delivery		< 0.001			
Very preterm (reference)					
Late preterm	3.023	< 0.001	20.562	4.686	90.224
Term	4.080	0.002	59.155	4.508	776.241
Constant	-2.886	< 0.001	0.056		

The article "Tranexamic Acid in Pregnant Women With Placenta Previa: A Double-Blind, Multicenter Randomized Clinical Trial" was retracted in 2025. Reasons: original data or images not available; unreliable results or conclusions; concerns about the article.

## Discussion

The findings of this study revealed that TXA was significantly more effective than the placebo in managing vaginal bleeding due to placenta previa, highlighting the potential efficacy of TXA as a targeted intervention in this high-risk population.

The cessation of vaginal bleeding in the intervention group may be attributed to specific mechanisms underlying TXA action. TXA is a synthetic lysine analog that binds to plasminogen and reduces the binding of plasminogen to fibrin, thereby inhibiting fibrinolysis. Therefore, it is frequently used for maintaining hemostasis and reducing blood loss [23]. Clinically, significant bleeding can occur due to surgery, trauma, obstetric complications, or various hemostatic disorders. As the causes of bleeding are diverse and not always immediately apparent, the availability of a safe, effective, and nonspecific hemostatic agent is critical in a wide range of clinical situations. Notably, antifibrinolytic agents are often used for this purpose [11]. Similarly, recurrent painless vaginal bleeding is the main symptom of placenta previa, and TXA treatment decreases vaginal blood loss.

The current study revealed that the rate of term pregnancies in the TXA group was significantly higher than that in the placebo group, with a greater difference in the rate of prolonged pregnancy from the time of first admission, receiving TXA, and delivery age. Women with placenta previa who present with antepartum bleeding have higher rates of preterm uterine contractions and preterm deliveries [9,24].

A reduction in preterm labor rates was associated with improved perinatal outcomes in the TXA group compared with the placebo group. Preterm delivery is a well-known outcome of placenta previa and is accompanied by diverse perinatal outcomes, including early neonatal death, admission to the NICU, and low birth weight [6,25,26].

The placebo group required more hospital admissions for blood transfusions and packed red blood cell (PRBC) transfusions compared to the TXA group. TXA is a well-established treatment to reduce blood loss in various medical and surgical conditions, including cesarean section [27] and postpartum hemorrhage [28].

Most participants in this study underwent an elective and emergency CS due to placenta previa. This trend is reflective of the concern for risk to the mother and/or fetus necessitating emergency CS at any gestational age or planned CS at a gestational age of 38 weeks. This also highlights the infrequency of vaginal delivery, which occurred in only 4.8% of cases. Vaginal deliveries were selected based on criteria such as marginal placenta previa, fetal situation (including stillbirths), and general condition of the mother permitting this mode of delivery. These findings underscore the necessity of individualized treatment for each woman with placenta previa, considering not only the gestational age of the fetus but also other relevant factors. 

The article "Tranexamic Acid in Pregnant Women With Placenta Previa: A Double-Blind, Multicenter Randomized Clinical Trial" was retracted in 2025. Reasons: original data or images not available; unreliable results or conclusions; concerns about the article.

In the TXA group, no significant association was observed between the grades of placenta previa and bleeding outcomes. This indicates that all types of placenta previa exhibited similar responses to TXA in terms of decreased blood loss, prolonged pregnancy, and perinatal outcomes. In addition to TXA, normal or overweight BMI and late preterm to term delivery were significantly associated with the cessation of bleeding due to placenta previa. The potential link between decreased BMI and decreased vaginal bleeding is intriguing and warrants further attention. In this context, a larger body size could influence bleeding tendencies in women with placenta previa. Brittany et al. reported an association of increased pre-pregnancy BMI with increased maternal morbidity and bleeding among women with placenta previa [29]. Collectively, these findings highlight the importance of planning and prenatal care in women with placenta previa. Moreover, the association indicating that bleeding cessation is more likely to occur with a late-preterm birth rather than an earlier preterm delivery demonstrates the crucial role of this factor in the onset and progression of placenta previa and indicates the involvement of novel pathways, which should be explored in future studies.

Study strengths

The randomized, double-blind design of this study contributed to controlling the effects of confounding variables. Furthermore, our results can be generalized to a broader patient population, as we included participants from different geographic locations and from five teaching hospitals.

Literature on medical interventions for vaginal bleeding management strategies during pregnancy in women with placenta previa is lacking. Therefore, this is the first study to address this critical clinical issue. Nevertheless, large-scale multicenter trials are imperative to generalize these results. Additionally, further research in diverse healthcare settings is crucial to validate our findings and improve management strategies for women with placenta previa.

The article "Tranexamic Acid in Pregnant Women With Placenta Previa: A Double-Blind, Multicenter Randomized Clinical Trial" was retracted in 2025. Reasons: original data or images not available; unreliable results or conclusions; concerns about the article.

A key strength of this study was the use of TXA, an easily available and inexpensive drug with a favorable safety profile in obstetrics, ensuring the feasibility and generalizability of the study [11,12,30].

Study limitations

Although the multicenter design is a strength, heterogeneity in patient characteristics and clinical practices at the centers could influence study outcomes. Therefore, studies with larger sample sizes and wider enrollment areas are required to further explore the generalizability of our findings.

Furthermore, the lack of data on maternal outcomes specific to placenta previa was also the limitation of the study; however, this was not the aim of the present study. Importantly, no cases of maternal morbidity or mortality were reported in this study. Notably, women with hemodynamic instability and placenta accreta spectrum disorders were excluded from the study, which may have reduced the risk of poor maternal outcomes.

A major challenge of this study was the lack of literature on the efficacy of TXA for placenta previa during pregnancy, which restricted the availability of comparative data to apply the current findings to a broader evidence-based setting.

## Conclusions

This study provides compelling evidence that TXA intervention during pregnancy in women with placenta previa significantly outperforms other treatments in managing vaginal bleeding, prolonging pregnancy to a favorable gestational age, and improving neonatal outcomes. Therefore, we recommend conservative and individualized risk-benefit assessments that prioritize maternal and fetal safety. Large-scale studies with a significantly larger sample size may enhance the generalizability of the current findings and contribute to a comprehensive understanding of the role of TXA in improving perinatal outcomes.
